# Regulatory Mechanism of MicroRNA-9 / Long Non-Coding RNA XIST Expression on Mouse Macrophage RAW264.7 Apoptosis Induced by Oxidized Low Density Lipoprotein

**DOI:** 10.1080/21655979.2021.2018978

**Published:** 2022-02-02

**Authors:** Xiaoling Zhang, Si Wang, Yuyan Cai, Weihong He, Qing Yang, Chen Li

**Affiliations:** a Department of Cardiology, West China Hospital, Sichuan University, Chengdu, Sichuan Province, China; b Department of Physiology, West China School of Basic Medical Sciences and Forensic Medicine, Sichuan University, Chengdu, Sichuan Province, China; c Department of Animal Imaging Platform of Public Experimental Technology Center, West China Hospital of Sichuan University, Chengdu, Sichuan Province, China

**Keywords:** MiR-9, lncRNA XIST, macrophages, apoptosis, proliferation

## Abstract

It aims to analyze the influential mechanism of microRNA-9 (miR-9) and long non-coding RNA XIST (lncRNA XIST) expression on the proliferation and apoptosis of macrophages induced by oxidized-low density lipoprotein (ox-LDL). Firstly, lncRNA XIST overexpression vector was constructed, and then RAW264.7 cells were used as the research object. Methylthiazolyl tetrazolium (MTT) method, flow cytometry, and Western blot were used to detect and compare the differences of cell proliferation, apoptosis, and the expression levels of apoptosis signal-regulating kinase 1 (ASK1), c-Jun N-terminal kinase (JNK), matrix metalloproteinase-9 (MMP-9), and B-cell lymphoma-2 (Bcl-2) after ox-LDL induction and transfection of miR-9 mimic, miR-9 inhibitor and XIST expression vector, respectively. The results showed that lncRNA XIST overexpression vector was successfully constructed and transfected into cells, wh5ich can inhibit the expression level of miR-9. Compared with the normal control group, ox-LDL can inhibit cell proliferation, promote cell apoptosis, and increase the expression level of target protein. Moreover, transfection of XIST expression vector based on ox-LDL induction can significantly enhance the inhibition of cell proliferation, and promote cell apoptosis and the expression of target protein. Transfection of miR-9 mimic can improve the biological changes induced by ox-LDL. After co-transfection of miR-9 mimic and XIST expression vector based on ox-LDL induction, cell proliferation, apoptosis, and target protein expression level were not significantly different from those induced by ox-LDL alone. In summary, the increased expression level of miR-9 can inhibit the apoptosis of macrophages induced by ox-LDL. lncRNA XIST can positively regulate the apoptosis of macrophages induced by ox-LDL.

## 1. Introduction

Cardiovascular disease caused by atherosclerosis has seriously threatened people’s life and health. The main pathological change of atherosclerosis is the formation of plaque, and the stability of plaque can directly affect the development of acute coronary syndrome [1]. The main pathological change of intimal plaque formation in atherosclerosis is the chronic inflammatory reaction of arteries, so oxidized-low density lipoprotein (ox-LDL) plays an important role in the occurrence and development of the disease [2]. Macrophages can form foam cells by phagocytosis of excess ox-LDL. These foam cells will form atheromatous necrosis after necrosis, eventually leading to the formation of atherosclerotic plaques [3]. Therefore, in the process of atherosclerosis, the number of macrophages and neovascularization can directly determine the stability of plaque.

Macrophage apoptosis is a chronic cumulative response, and there are many factors that promote macrophage apoptosis, such as ox-LDL, oxidative stress response, and some cytokines [4,5]. With the rapid development of transcriptome sequencing technology, a large number of studies indicated that microRNA (miRNA) and long non-coding RNA (lncRNA) can participate in the whole cell biological process as regulatory factors, and play a promoting or inhibiting role in many diseases [6]. Studies confirmed that miR-9 can promote the apoptosis of myocardial cells, and then play an important role in myocardial remodeling after myocardial infarction [7]. LncRNA XIST gene is located in human chromosome Xq13.2, and it can participate in and regulate the inactivation of X chromosome. In addition, many studies confirmed that XIST gene can participate in many cancer processes, such as breast cancer, ovarian cancer, and lung cancer [8–10]. lncRNA XIST can regulate the osteogenic differentiation of human bone marrow stromal cells (hBMSCs) by regulating miR-9-5p [11].

It plays an important role in the formation of arteriosclerosis, upregulating the expression of miR-9 can inhibit macrophages to form foam cells, lncRNA XIST can regulate the polarization of macrophages, the combination of the two can regulate the proliferation and apoptosis of macrophages, which has a regulatory role in atherosclerotic diseases. However, the mechanism of lncRNA XIST and miR-9 in atherosclerosis is still unclear. Drawing on experience from previous research results, it was speculated that elevated miR-9 expression level was able to inhibit ox-LDL inducing macrophage apoptosis. LncRNA XIST can positively regulate ox-LDL inducing macrophage apoptosis. Thus, ox-LDL was first used to induce apoptosis of macrophages in this research, and then miR-9 and lncRNA XIST were transfected to analyze their effects on cell proliferation and apoptosis. The purpose of this research was providing new ideas for the stability of atherosclerotic plaque and the prevention and treatment of acute coronary syndrome to investigate the regulatory mechanism of miR-9 and lncRNA XIST expression on ox-LDL-induced apoptosis in macrophages.

## 2. Materials And Methods

### 2.1 Materials

Dulbecco’s Modified Eagles Medium (DMEM), fetal bovine serum, and Opti-MEM were all purchased from Gibco of the United States. miR-9 mimic and inhibitor were purchased from Shanghai GenePharma Co.,Ltd. pcDNA3.1 carrier and Lipofectamine 2000 were purchased from Invitrogen of the United States. Methylthiazolyl tetrazolium (MTT) kit was purchased from Sigma of the United States. SYBR green PCR kit and cDNA reverse transcription kit were all purchased from Takara of Japan. Dimethyl sulfoxide (DMSO), bicinchoninic acid (BCA) protein detection kit, and poly (vinylidene fluoride) (PVDF) were all purchased from Shanghai Beyotime Biotechnology. ECL luminescent detection kit was purchased from Thermo fisher of the United States. Both protein primary antibody and secondary antibody were purchased from Abcam of the UK.

### 2.2 Culture of RAW264.7 cells

RAW264.7 cells were cultured in high glucose DMEM medium containing 10% fetal bovine serum and cultured in a 37°C-incubator containing 5% CO_2_ for 2 days to observe the cell state. When the cell confluence reached about 80%, the cell culture medium was replaced and the cell passage was processed, and the passage ratio was 1:4. All the subsequent experiments were performed with the cells in logarithmic growth stage.

### 2.3 Cell transfection of miR-9 mimic and inhibitor

RAW264.7 cells were inoculated in 96-well plates and medium, and cells were starved by the supplemented Opti-MEM medium without double antibody for 12 h. The miR-9 mimic, miR-9 inhibitor, and Lipofectamine 2000 reagents were diluted in Opti-MEM medium without double antibody, and then they were allowed to stand for 5 min at room temperature and mixed well. After 20 minutes, Opti-MEM medium was added to adjust the final concentration of miR-9 mimic and miR-9 inhibitor to 50 nM and 100 nM, respectively, and RNA-liposome mixture was added dropwise. The original medium in each well of RAW264.7 cells was discarded, mixed transfection solution was added dropwise, and the cells were cultured in a cell incubator for further culture for 6 h. The original culture medium was discarded, the normal cell medium was added for further culture for 48 h, and the cells were collected for detection.

### 2.4 Cell transfection of lncRNA XIST

The amplification primers of lncRNA XIST (F: 5ʹ-GTCCCCCAGCAGGCTTTATC-3ʹ; R: 5ʹ-GAAAAGTGAGTGAAGGAGTA-3ʹ) were designed, which was ligated into pcDNA3.1 expression vector. After double enzyme digestion and sequencing, the overexpression plasmid was transfected with Lipofectamine 2000 reagent. The procedure of transfection was the same as section 2.2.3.

### 2.5 Cell grouping

According to the experimental treatment method, RAW264.7 cells were divided into 9 groups, which were as follows: (1) control group, i.e. normal RAW264.7 cells without any treatment; (2) ox-LDL group, i.e. 100 μg/mL ox-LDL was used for the induction of RAW264.7 cells; (3) miR-9 mimic group, no ox-LDL induction for miR-9 mimic transfection; (4) miR-9 inhibitor group, no ox-LDL induction for miR-9 inhibitor transfection; (5) XIST group, no ox-LDL induction for lncRNA XIST expression vector transfection; (6) miR-9 mimic + ox-LDL group, miR-9 mimic transfection on the basis of 100 μg/mL ox-LDL induction treatment; (7) miR-9 inhibitor + ox-LDL group, miR-9 inhibitor transfection on the basis of 100 μg/mL ox-LDL induction treatment; (8) XIST + ox-LDL group, lncRNA XIST expression vector transfection on the basis of 100 μg/mL ox-LDL induction treatment; (9) miR-9 mimic+XIST group, miR-9 mimic and lncRNA XIST expression vectors were transfected based on 100 μg/mL ox-LDL induction [12].

### 2.6 MTT assay for detection of cell proliferation activity

The cells in each group were collected after 48 h of treatment, and 20 μL 5 mg/mL MTT solution was added to each well for further culture for 4 h. The original medium was discarded, and 150 μL DMSO solution was added to each well, blended gently for 10 min. Finally, the absorbance of cells in each well was detected at 490 nm by enzyme-labeled instrument. The cell activity was calculated by comparing the cells absorbance of the control group and the experimental group [13].

### 2.7 Detection of apoptosis by flow cytometry

Phosphate-buffered saline (PBS) was prepared into 75% ethanol solution using precooled anhydrous ethanol solution. Cells in each group were collected after 48 h of treatment and washed with precooled PBS. Cells were digested with 0.25% trypsin, and the normal medium was added to prepare cell suspension, which was centrifuged at 1000 rpm for 5 min. The supernatant was discarded, and then precooled PBS was added to resuspend cells for cell washing. Then, the Annexin V/PI kit was used to stain the cells, and the apoptosis was detected [14].

### 2.8 RT-PCR

Precooled Trizol solution was used for the extraction of total RNA from cells, and the concentration and purity of total RNA were detected. lncRNA XIST or miR-9 RT primer was added, and the cDNA was reverse transcribed by RT kit. Subsequently, the target gene was amplified according to the reaction system in the instructions of the fluorescent quantitative PCR detection kit. The amplification procedure of lncRNA XIST was as follows: 95°C (60s), 95°C (15s), 60°C (60s), 72°C (30s), 40 cycles. In the amplification primer information, the upstream primer was as follows: 5ʹ-GCATAACTCGGCTTAGGGCT-3ʹ, and the downstream primer was as follows: 5ʹ-TCCTCTGCCTGACCTGCTAT-3ʹ. The amplification procedure of miR-9 was as follows: 94°C (10 min), 94°C (15s), 65°C (60s), 72°C (30s), 40 cycles. The amplification primer information was as follows: 5ʹ-UCUUUGGUUAUCUAGAUGUAUGA-3ʹ. β-actin was used as the reference gene, and in the amplification primer information, the upstream primer was as follows: 5ʹ- TGTGGGCATCAATGGATTTGG-3ʹ, and the downstream primer was as follows: 5ʹ- ACACCATGTATTCCGGGTCAAT-3ʹ. Finally, the relative expression quantity of lncRNA XIST and miR-9 was calculated by 2^−ΔΔCt^ method.

### 2.9 Western blot

RIPA was used for the extraction of total cellular proteins, and BCA protein detection kit was used for the quantification of protein concentration. Subsequently, 25 mg protein was taken and 10% SDS-PAGE gel was prepared for electrophoresis separation. The separated protein was transferred to PVDF membrane and sealed with 5% skim milk for 1 h. Then, ASK1 (1:1500), JNK (1:1500), MMP-9 (1:1500), Bcl-2 (1:1500), and β-actin (1:2000) monoclonal primary antibody were used for overnight incubation of the sample in the 4°C refrigerator. Subsequently, the horseradish peroxidase-labeled anti-rabbit secondary antibody (1:800) was used to incubate the sample for 2 h at room temperature. Finally, ECL luminescence kit was used to dye the target protein band for 2 min, and that was placed in a gel imager for development and fixation.

### 2.10 Statistical processing

SPSS19.0 software was used for statistical analysis. All experimental data were expressed as mean ± standard deviation (x̅ ± s) and the differences among groups were compared by independent sample *t* test or single factor ANOVA. The relative expression quantity of target gene was calculated by 2^−ΔΔCt^ method. *P* < 0.05 was considered statistically significant.

## 3. Results

In this study, it mainly investigated the regulatory mechanism of miR-9 and lncRNA XIST expression on ox-LDL-induced macrophage apoptosis, successfully constructed lncRNA XIST overexpression vector, transfected it into cells, detected cell proliferation activity by MTT assay, detected apoptosis by flow cytometry, detected the expression levels of miR-9 and lncRNA XIST, analyzed the effects of the two on apoptosis and proliferation, and investigated the effects of miR-9 and lncRNA XIST on the expression of target proteins in cells.

### 3.1 Detection of miR-9 expression level

The difference of miR-9 expression levels among groups was detected by RT-PCR, as shown in Figure 1. Compared with the normal control group, the expression levels of miR-9 in the cells were significantly decreased after the addition of ox-LDL, ox-LDL + miR-9 inhibitor, and ox-LDL + lncRNA XIST. The difference was statistically significant (*P* < 0.05). After the addition of ox-LDL + miR-9 mimic, the expression level of miR-9 in cells was significantly increased, and the difference was statistically significant (*P* < 0.05). However, there was no significant difference in miR-9 expression level between normal control group and cells added with ox-LDL + miR-9 mimic + lncRNA XIST (*P* > 0.05).

**Figure 1.** The difference of miR-9 expression level in cells among groups (* *P* < 0.05).

### 3.2 Detection of lncRNA XIST expression level

RT-PCR was used to detect the difference in the expression level of lncRNA XIST in cells among groups, as shown in Figure 2. Compared with the normal control group, the expression levels of lncRNA XIST in the cells were significantly increased after the addition of ox-LDL, ox-LDL + miR-9 inhibitor, and ox-LDL + lncRNA XIST. The difference was statistically significant (*P* < 0.05). After addition of ox-LDL + miR-9 mimic, the expression level of lncRNA XIST in cells was significantly decreased, and the difference was statistically significant (*P* < 0.05). However, there was no significant difference in lncRNA XIST expression level between normal control group and cells added with ox-LDL + miR-9 mimic + lncRNA XIST (*P* > 0.05).

**Figure 2.** The difference of lncRNA XIST expression level in cells among groups (* *P* < 0.05).

### 3.3 Effects of miR-9 and lncRNA XIST on cell proliferation

MTT was used to detect the difference of cell absorbance at 6 h, 12 h, 24 h, and 48 h after treatment. The results are shown in Figure 3. Figure 3a shows that compared with the normal control group, ox-LDL, and ox-LDL + miR-9 mimic treatment group, the cell proliferation activity was significantly decreased after addition of ox-LDL + miR-9 inhibitor, ox-LDL + lncRNA XIST, and ox-LDL + miR-9 + lncRNA XIST 6 h after treatment, and the difference was statistically significant (*P* < 0.05).**Figure 3.** Changes of cells proliferation activity in groups at different treatment time (Figure A was 6 h after treatment. Figure B was 12 h after treatment. Figure C was 24 h after treatment. Figure D was 48 h after treatment. Compared with normal control group, * *P* < 0.05. Compared with ox-LDL, # *P* < 0.05. Compared with ox-LDL + miR-9 mimic, & *P* < 0.05. Compared with ox-LDL + lncRNA XIST, ^ *P* < 0.05).

**Figure 3.** Continued.

Figure 3b-3d shows that compared with the normal control group, the cell proliferation activity of other groups was significantly decreased, and the difference was statistically significant (*P* < 0.05) 12 h, 24 h, and 48 h after treatment. Compared with ox-LDL group, the addition of miR-9 mimic can significantly increase the proliferation activity of cells, and the difference was statistically significant (*P* < 0.05). However, the proliferation activity of cells after addition of miR-9 inhibitor and lncRNA XIST decreased significantly, and the difference was statistically significant (*P* < 0.05). However, there was no significant change in cell proliferation activity after adding miR-9 mimic + lncRNA XIST at the same time (*P* > 0.05). Compared with ox-LDL + lncRNA XIST group, addition of miR-9 mimic can significantly increase the proliferation activity of cells, and the difference was statistically significant (*P* < 0.05).

### 3.4 Effects of miR-9 and lncRNA XIST on apoptosis

Annexin V-FTIC/PI was used to detect apoptosis. The results are shown in Figure 4. lncRNA XIST can significantly promote the apoptosis of cells, and addition of miR-9 mimic can inhibit the apoptosis caused by lncRNA XIST.

**Figure 4.** Annexin V-FTIC/PI staining of apoptosis in all groups (× 200).

The differences among apoptosis rates of all groups were measured by flow cytometry, and the results are shown in Figure 5. Compared with the normal control group, the addition of ox-LDL, ox-LDL + miR-9 inhibitor, ox-LDL + lncRNA XIST, and ox-LDL + miR-9 mimic + lncRNA XIST can significantly increase the apoptosis rate of the cells, and the difference was statistically significant (*P* < 0.05). However, there was no significant difference in apoptosis rate between the normal control group and ox-LDL + miR-9 mimic group (*P* > 0.05). Compared with ox-LDL group, addition of miR-9 mimic can significantly reduce the apoptosis rate, and the difference was statistically significant (*P* < 0.05). However, addition of miR-9 inhibitor and lncRNA XIST based on ox-LDL can significantly increase the apoptosis rate, and the difference was statistically significant (*P* < 0.05), and the apoptosis rate of lncRNA XIST was more obvious. Compared with ox-LDL + lncRNA XIST, addition of miR-9 mimic can significantly reduce the apoptosis rate, and the difference was statistically significant (*P* < 0.05).

**Figure 5.** Comparison of apoptosis rates among groups. (Compared with the normal control, * *P* < 0.05. Compared with ox-LDL, # *P* < 0.05. Compared with ox-LDL + miR-9 mimic, & *P* < 0.05. Compared with ox + LDL + miR-9 inhibitor, @ *P* < 0.05. Compared with ox-LDL + lncRNA XIST, ^ *P* < 0.05).

### 3.5 Effects of miR-9 and lncRNA XIST on target protein expression of cells

The differences in ASK1, JNK, MMP-9, and Bcl-2 protein levels among groups were detected by Western blot, and the results are shown in Figure 6. Compared with the normal control group, adding ox-LDL, ox-LDL + miR-9 inhibitor, ox-LDL + lncRNA XIST, and ox-LDL + miR-9 mimic + lncRNA XIST increased the relative expression levels of ASK1, JNK, MMP-9, and Bcl-2 protein in cells, and the differences were statistically significant (*P* < 0.05). Compared with ox-LDL, addition of miR-9 mimic reduced the expression of the target protein, while the addition of miR-9 inhibitor and lncRNA XIST reduced the expression of the target protein, and the difference was statistically significant (*P* < 0.05). Compared with ox-LDL + lncRNA XIST, the expression level of target protein in cells decreased significantly after addition of miR-9 mimic, and the difference was statistically significant (*P* < 0.05).

**Figure 6.** Comparison of the relative expression of the target protein of cells among groups. (Figure A was the Western blot strip. Figure B was the relative expression quantity of ASK1. Figure C was the relative expression quantity of JNK. Figure D was the relative expression quantity of MMP-9. Figure E was the relative expression quantity of Bcl-2. Compared with normal control, * *P* < 0.05. Compared with ox-LDL, # *P* < 0.05. Compared with ox-LDL + miR-9 mimic, & *P* < 0.05. Compared with ox + LDL + miR-9 inhibitor, @ *P* < 0.05. Compared with ox-LDL + lncRNA XIST, ^ *P* < 0.05).

**Figure 6.** Continued.

**Figure 6.** Continued.

## 4. Discussion

Apoptosis of macrophage-derived foam cells is a major feature of advanced atherosclerosis. In the lesions of advanced atherosclerosis, the necrosis core caused by macrophage apoptosis can promote the rupture of plaque, and eventually lead to vascular occlusion and tissue infarction [15]. Therefore, it is of great significance to analyze the apoptosis mechanism of macrophages in the process of atherosclerosis for understanding the occurrence and development of the disease. There are many factors leading to macrophage apoptosis, among which the accumulation of lipids and cholesteryl esters are the reasons leading to macrophage apoptosis and affecting plaque stability [16,17]. As a regulatory molecule, miRNAs have a variety of regulatory effects on macrophages, which can produce pro-inflammatory cytokines. Studies found that miRNAs can regulate the inflammatory response and affect the production of cytokines by macrophages, and some miRNAs can also regulate the phagocytosis of macrophages. Therefore, ox-LDL was used to induce RAW264.7 macrophages to construct the model in this research. The results showed that compared with normal RAW264.7 cells, the proliferation activity of cells induced by ox-LDL decreased significantly, and the apoptosis rate increased significantly. These results indicated that the macrophage apoptosis model was successfully constructed by ox-LDL, which laid a foundation for further research.

miRNA is an endogenous non-coding small RNA with regulatory effect in eukaryotic cells, which can participate in the expression of all genes in eukaryotic cells. Studies indicated that miRNA is only expressed in specific tissues or developmental stages, and plays an important regulatory role in cell growth and development [18]. miRNA-9 is abundant in brain tissue, and studies showed that it can participate in the proliferation and differentiation of neural stem cells [19]. However, studies confirmed that miRNA-9 plays an important role in the process of atherosclerosis [20]. Shao et al. (2020) [21] confirmed that anthocyanin can inhibit the apoptosis of macrophages caused by ox-LDL, and anthocyanin can inhibit the formation of foam cells by macrophages by up-regulating the expression of miR-9. Studies found that ox-LDL can induce macrophage-derived foam cells and alleviate atherosclerosis [22]. In this study, miR-9 was transfected to further explore its regulatory mechanism. In this research, miRNA-9 mimic and its inhibitor were transfected into ox-LDL-induced macrophages, and the results showed that miRNA-9 mimic can improve the apoptosis induced by ox-LDL. It was indicated that the up-regulation of miR-9 can inhibit the apoptosis of macrophage-derived foam cells, thereby improving the process of atherosclerosis.

lncRNA can participate in the regulation of gene transcription, protein activity, chromosome structure remodeling, and other cell biological processes. lncRNA XIST was first found to be able to participate in the initiation stage of X chromosome inactivation, and it can participate in the process of various cancer diseases, and affect the proliferation and invasion of tumor cells [23,24]. The research suggested that lncRNA XIST can regulate the expression of TCF-4, and then regulate the polarization of macrophages in lung cancer [25]. In addition, it is confirmed that lncRNA XIST can participate in the regulation of the toxic effect of M1 macrophages on chondrocytes in osteoarthritis [26]. Therefore, it is supposed that lncRNA XIST can play an important role in atherosclerosis by participating in the biological process of macrophage regulation. The expression vector of XIST was prepared and transfected into ox-LDL-induced apoptosis model of macrophages. The results showed that XIST can aggravate the apoptosis of macrophages.

To explore the effect of miR-9 and lncRNA XIST on macrophage apoptosis, this research co-transfected miR-9 mimic and XIST expression vector into ox-LDL-induced macrophage apoptosis model. The results showed that upregulation of miR-9 expression can neutralize the effect of XIST on macrophage apoptosis. To further explore the mechanism of miR-9 and lncRNA XIST regulating the apoptosis of macrophages, the expression levels of ASK1, JNK, MMP-9, and Bcl-2 were detected. ASK1-JNK pathway is involved in the regulation of apoptosis [27]. MMP-9 protein can participate in the angiopoietic process by releasing vascular endothelial growth factor [28]. Bcl-2 protein belongs to the coding product of proto-oncogene Bcl-2, which can participate in the regulation of apoptosis [29]. These four proteins are important in the regulation of apoptosis. The results showed that compared with ox-LDL-induced macrophage apoptosis, transfection of miR-9 mimic can inhibit the expression of ASK1, JNK, MMP-9, and Bcl-2 protein, while transfection of XIST expression vector can promote the expression of ASK1, JNK, MMP-9, and Bcl-2 protein. Co-transfection of miR-9 mimic and XIST expression vector can maintain the expression balance of ASK1, JNK, MMP-9, and Bcl-2 protein. The apoptosis rate was the highest in the XIST group, but the expression level of Bcl-2 protein was the highest, which may be the counteraction of Bax factor, Bcl-2 has an anti-apoptotic effect, and Bax can promote apoptosis.

## 5. Conclusion

In conclusion, miR-9 and lncRNA XIST can participate in the process of macrophage apoptosis induced by ox-LDL, and the regulation may be realized through ASK1-JNK pathway. This research only compared the mechanism of miR-9 and lncRNA XIST expression changes on ox-LDL-induced macrophage proliferation and apoptosis, and did not verify whether lncRNA XIST can directly regulate miR-9 expression. Therefore, it is necessary to use dual-luciferase reporter gene to analyze the binding targets of lncRNA XIST and miR-9, predict the target genes of miR-9, and analyze the development mechanism of atherosclerosis at the lncRNA-miRNA-mRNA level. In summary, the results of this research can provide a reference for understanding the process of atherosclerosis.

## Highlights

- miR-9 is up-regulated and can inhibit apoptosis of macrophage foam cells.
- LncRNA XIST can exacerbate apoptosis in macrophages.
- miR-9 can inhibit the expression of ASK1, JNK, MMP-9, and Bcl-2 protein.
- LncRNA XIST can promote the expression of ASK1, JNK, MMP-9, and Bcl-2 protein.
